The article "Repressing phosphatidylinositol-4,5-bisphosphate 3-kinase catalytic subunit gamma by microRNA-142-3p restrains the progression of hepatocellular carcinoma" was retracted in 2024. Reasons: original data or images not available; unreliable results or conclusions; concerns about the data; concerns about the results or conclusions.

# Repressing phosphatidylinositol-4,5-bisphosphate 3-kinase catalytic subunit gamma by microRNA-142-3p restrains the progression of hepatocellular carcinoma

**DOI:** 10.1080/21655979.2021.2020549

**Published:** 2022-01-06

**Authors:** Chuanli Zeng, Gang Yuan, Yaoren Hu, Donghui Wang, Xiaojun Shi, Dedong Zhu, Airong Hu, Yina Meng, Jialin Lu

**Affiliations:** a Department of Severe Liver Disease, Ningbo HuaMei Hospital, University of Chinese Academy of Science, Ningbo, Zhejiang, China; b Department of Acute Infection, Ningbo Huamei Hospital, University of Chinese Academy of Science, Ningbo, Zhejiang, China; c Ningbo Institute of Life and Health Industry, University of Chinese Academy of Science, Ningbo, Zhejiang, China; d Key Laboratory of Diagnosis and Treatment of Digestive System, Tumors of Zhejiang Province, China; e Department of Hepatology, Ningbo Huamei Hospital, University of Chinese Academy of Science, Ningbo, Zhejiang, China; f Institute of Liver Disease, Ningbo Huamei Hospital, University of Chinese Academy of Sciences, Ningbo, Zhejiang, China; g Medical School of Ningbo University, Ningbo, Zhejiang, China

**Keywords:** Mir-142-3p, pik3cg, hepatocellular carcinoma, apoptosis

## Abstract

This paper probes the mechanisms underlying miR-142-3p’s modulation of hepatocellular carcinoma (HCC) invasion and apoptosis. Quantitative real-time PCR and Western blot monitored the miR-142-3p profile in HCC tissues and non-tumor tissues. The correlation between miR-142-3p expression and HCC patients’ clinicopathological indicators was analyzed. miR-142-3p overexpression and knockdown models were established in HCC cell lines. Cell proliferation was gauged by the colony formation assay and BrdU staining. For measuring apoptosis, flow cytometry and Western blot were implemented. Transwell assay tested cell migration and invasion. miR-142-3p mimics or inhibitors were transfected in Huh7 and HCCLM3 cells. The targeting association between miR-142-3p and PIK3CG was predicted through bioinformatics and further verified by related experiments. The influence of PIK3CG overexpression on miR-142-3p’s role in HCC was assayed. A xenografted tumor model was built in mice to validate miR-142-3p knockdown’s influence on HCC *in vivo*. As a result, miR-142-3p exhibited a decreased profile in HCC tissues and cells. Overexpressing miR-142-3p accelerated apoptosis and suppressed the PI3K/AKT/HIF-1α signal. Knocking down miR-142-3p presented opposite effects. PIK3CG overexpression dampened the anti-tumor effect of miR-142-3p. miR-142-3p repressed HCC invasion and intensified apoptosis to restrain HCC by abating the PIK3CG-mediated PI3K/AKT/HIF-1α pathway.

## Introduction

Hepatocellular carcinoma (HCC), a familiar malignancy, is a prime contributor to cancer-associated deaths in the world [1]. HCC is widespread in China on account of the prevalence of the hepatitis B virus [2]. Ultrasonography (US) and alpha-fetoprotein (AFP) tests are universal screening methods for high-risk groups. Nevertheless, because of the poor effectiveness of the AFP test and the high reliance of the US on the operator, the effect of the early screening and diagnosis is not satisfactory [3]. Clinically, surgical resection and liver transplantation are the most frequent treatments for HCC. However, the high recurrence rate and high metastasis rate reveals the suboptimal clinical effectiveness [4]. Therefore, the major problems for treating HCC are the difficulty of early diagnosis and the high rate of recurrence and metastasis, and identifying new types and effective treatment targets for HCC is critically significant.

The article "Repressing phosphatidylinositol-4,5-bisphosphate 3-kinase catalytic subunit gamma by microRNA-142-3p restrains the progression of hepatocellular carcinoma" was retracted in 2024. Reasons: original data or images not available; unreliable results or conclusions; concerns about the data; concerns about the results or conclusions.

MicroRNAs (miRNAs) are evolutionarily conserved non-coding RNAs composed of 18–25 nucleotides [5]. In recent years, miR-142-3p, as a crucial miRNA, has received accumulating attention due to its potential appliance in HCC diagnosis and treatment. For example, some researchers elucidate that circRNA WHSC1 (CircWHSC1), an oncogene, motivates homeobox A1 (HOXA1) expression by sponging miR-142-3p, therefore exerting carcinogenic roles in HCC [6]. Moreover, miR-142-3p expression presents a dramatic diminution in HCC. Long non-coding RNA Lnc712 (LncRNA712) targets the miR-142-3p/Bach-1 pathway, thus facilitating HCC development [7]. The research by Yu Q et al. has manifested that miR-142-3p represses HCC proliferation, migration, and epithelial-mesenchymal transition (EMT). Metastasis-associated lung adenocarcinoma transcript 1 (MALAT1), a competing endogenous RNA, accelerates HCC progression through the sponge of miR-142-3p expression [8]. More importantly, Fu Y et al. have initially reported that miR-142-3p, a novel tumor suppressor, impedes HCC cell invasion and migration by directly modulating the high mobility group box protein 1 (HMGB1) transcription [9]. Hence, miR-142-3p shows outstanding values in suppressing HCC development. However, whether miR-142-3p influences the biological behaviors of HCC through other mechanisms of action is not well characterized.

The phosphatidylinositol 3-kinase (PI3K)/AKT pathway contributes to various cellular activities and pathological mechanisms as a classical signaling pathway. Hypoxia-inducible factor 1α (HIF-1α) is under the modulation of oxygen concentration as a nuclear transcription factor, with the specific activity under hypoxia [10]. Furthermore, HIF-1α, the PI3K/AKT signal’s downstream factor, is the initiator of the endogenous protect mechanism [11,12]. Studies have illuminated that Huaier restrains lung cancer cells’ growth, migration and energy metabolism via inactivation of PI3K/AKT/HIF-1α[13]. In parallel, epigallocatechin gallate derivative Y6 (EGCG Y6) chokes HCC angiogenesis through MAPK/ERK/2 and PI3K/AKT/HIF-1α/VEGF [14]. Additionally, Yu L et al. have manifested that Girdin regulates HCC glycolysis through the PI3K/AKT/HIF-1α axis, thus lowering HCC cells’ sensitivity to radiotherapy [15]. These data confirm that the PI3K/AKT/HIF-1α pathway exerts a momentous part in the glycolysis and angiogenesis of HCC. However, whether it has involvement in HCC proliferation, migration and invasion requires to be further probed.

The article "Repressing phosphatidylinositol-4,5-bisphosphate 3-kinase catalytic subunit gamma by microRNA-142-3p restrains the progression of hepatocellular carcinoma" was retracted in 2024. Reasons: original data or images not available; unreliable results or conclusions; concerns about the data; concerns about the results or conclusions.

PIK3CG is the sole member of the IB PI3K family, which contributes to diversified tumors. For instance, researchers reveal that PIK3CG presents high expression in prostate cancer, and inhibition of PIK3CG prevents prostate cancer growth and EMT to alleviate tumor metastasis *in vivo* [16]. Besides, Wang J et al. have discovered that knocking down microRNA-1976 (miR-1976) expedites EMT and cancer stem cell metastasis in triple-negative breast cancer by augmenting PIK3CG [17]. What’s more, Chen S et al. have elucidated that microRNA-502 (miR-502) dampens HCC progression by restraining PI3KCG [18]. The above evidence suggests that PI3KCG has associations with HCC progression. Nonetheless, whether miR-142-3p influences HCC’s biological behaviors through the modulation of PI3KCG remains elusive.

In this paper, the underlying role of miR-142-3p in HCC was investigated. As a result, miR-142-3p repressed HCC proliferation, migration, and invasion. Meanwhile, we observed that miR-142-3p reversely modulated PI3KCG profiles through suppression of the PI3K/AKT/HIF-1α signal. This freshly discovered miR-142-3p/PAX5/PI3KCG/AKT/HIF-1α signal may exert crucial properties in HCC evolution and metastasis. Therefore, the comprehension of the signal may favor seeking novel strategies for HCC treatment.

This research tested the miR-142-3p profile in HCC tissues and paracancerous non-tumor tissues and HCC cells. The outcomes revealed significant down-regulation of miR-142-3p in HCC tissues and cell lines. Notably, overexpressing miR-142-3p restrained HCC cell proliferation and fostered apoptosis. Bioinformatics analysis signified that PIK3CG was a downstream target of miR-142-3p. Knocking down miR-142-3p up-regulated PIK3CG and stimulated the PI3K/AKT/HIF-1α axis. Thus, we posited that miR-142-3p regulated HCC through targeted inhibition of PIK3CG. Overall, this study addresses the specific molecular mechanisms in modulating HCC progression, providing new targets and directions for HCC diagnosis and treatment.

The article "Repressing phosphatidylinositol-4,5-bisphosphate 3-kinase catalytic subunit gamma by microRNA-142-3p restrains the progression of hepatocellular carcinoma" was retracted in 2024. Reasons: original data or images not available; unreliable results or conclusions; concerns about the data; concerns about the results or conclusions.

## Materials and methods

### Collection and process of clinical specimens

Human HCC tissues and adjacent matched healthy tissues were acquired from 50 HCC patients who were subjected to hepatectomy in HuaMei Hospital of the University of Chinese Academy of Science from March 2016 to September 2018. The 50 patients had no previous history of malignancy and no other serious clinical conditions such as diabetes or heart disease. None of the patients received adjuvant therapy, such as chemotherapy or radiotherapy prior to the operation. The control specimens were acquired from the same patient’s paracancerous tissues (at least 3 cm from the surgical margin), and no tumor cells were observed in the postoperative pathological checking. The diagnosis of HCC was pathologically verified following the standards of the World Health Organization (WHO). Following the acquisition, all samples were rapidly preserved in liquid nitrogen at −196°C for extracting RNA. Our research met the approval of the research ethics committee of HuaMei Hospital of the University of Chinese Academy of Science. A written informed consent form was signed by all patients who agreed to the scientific application of the tissue collection before liver resection [7].

### Cell culture and transfection

We ordered HCC cell lines (HCCLM3 and Huh-7) and a hepatocellular cell line L-O2 from the American Type Culture Collection (Manassas, VA, USA). Dulbecco’s Modified Eagle’s medium (DMEM) comprising 10% fetal bovine serum (FBS, Gibco, Thermo Scientific, Shanghai, China), 100 U/mL penicillin, and 100 μg/mL streptomycin (Gibco, Thermo Scientific, Shanghai, China) was applied for cell growth. Then, cell culture was performed at 37°C with 5% CO_2_.

We obtained miR-142-3p mimics, negative controls (miR-NC), miR-142-3p inhibitors and their negative controls (miR-in) from GenePharma (Shanghai, China). Then, the pcDNA3.1-PIK3CG expression vector was built by embedding the overall length of PIK3CG cDNA into the backbone of the pcDNA3.1 vector. Next, the transfection was conducted by utilizing Lipofectamine 2000 (Invitrogen, Grand Island, NY, USA) as guided by the manufacturer. In short, the miRNA (50 nM) or plasmid (100 µg) undergoing dilution in 100 µL of OPTI-MEM (Thermo Scientific, Shanghai, China) was subjected to mix with 10 µL of lipofectamine for 15-minute incubation at room temperature (RT). Finally, 48 hours of culture was carried out after adding the mixture to the cells for further analysis [19].

### Colony formation assay

The inoculation of HCCLM3 and Huh-7 cells in the log phase was performed in 6-well plates (500 cells/well) for 8-day incubation. Subsequently, each well’s growth medium was substituted every 3 days. On completion of each experiment, 1 mL of 4% paraformaldehyde was employed for 30–60-minute fastening of the cells. Next, the cells rinsing with phosphate-buffered saline (PBS) underwent 10–20-minute immersion in 500 μL of Giemsa (AR-0752; Shanghai Dingguo Biotechnology Co., Ltd). A microscope was utilized for photographing and counting the cell colonies [20].

The article "Repressing phosphatidylinositol-4,5-bisphosphate 3-kinase catalytic subunit gamma by microRNA-142-3p restrains the progression of hepatocellular carcinoma" was retracted in 2024. Reasons: original data or images not available; unreliable results or conclusions; concerns about the data; concerns about the results or conclusions.

### BrdU experiment

10 μmol/L BrdU (Sigma, Shanghai, China) was added to HCCLM3 and Huh-7 cells in the log phase. After DNA denaturation, the cells underwent 2-hour incubation at RT with the BrdU primary antibody (Abcam, ab6326, 1:1000, CA, USA). Next, a fluorescent secondary antibody was affiliated to be incubated at RT for 2 hours. Afterward, 10 μmol/L Hoechst33342 was adopted to label the nucleus. Imaging and statistical analysis were carried out by applying an inverted fluorescence microscope [21].

### Transwell experiment

We employed Transwell chambers (Millipore, USA) to gauge cell migration and invasion. For the migration experiment, cells were grown with serum-free DMEM in the upper chamber, and the lower chamber was supplemented with 10% serum-containing DMEM. Cells were inoculated in the upper chamber containing the Matrigel-coated membrane at the bottom for the invasion assay. Following 24 hours of culture, 0.1% crystal violet was utilized to stain the migrated or invaded cells for 30 minutes. Experiments were conducted in triplicate [22].

### Flow cytometry (FCM)

The Annexin V-fluorescein isothiocyanate (AnnexinV-FITC) double staining method was taken for gauging cell apoptosis. Twenty-four hours following the transfection, the cells were trypsinized, harvested and seeded in 6-well plates (2 × 10^6^ cells/well). After 24-hour culture, we discarded the supernatant. Next, the cells were rinsed twice with pre-cooled PBS and resuspended in 1× Binding buffer. Afterward, 5 μL AnnexinV-FITC and 5 μL propidium iodide (PI) were spiked into the cell suspension for 15-minute incubation at RT after full stirring. Finally, FCM was implemented to assay the apoptotic rate within 1 hour under the kit instructions [22].

### Quantitative real-time PCR (qRT-PCR)

Total RNA was extracted out of cells by utilizing the TRIzol reagent (Invitrogen, Waltham, MA, USA). Subsequently, RNA underwent reverse transcription into cDNA utilizing the PrimeScript™ RT Reagent kit (Invitrogen, Shanghai, China). The Bio-Rad CFX96 quantitative PCR system and Synergy Brands (SYBR) were applied for implementing qRT-PCR, with pre-denaturation at 95°C for 5 minutes, denaturation at 95°C for 15 seconds, and annealing at 60°C for 30 seconds. U6 small nuclear RNA (U6) was the endogenous control of miR-142-3p. The relative expression was calculated with the 2^−∆∆Ct^ method [23]. miR-142-3p primers: forward 5’-GTCGTATCCAGTGCAGGG-3’, reverse 5’-CGACGTGTAGTGTTTCCTA-3’. U6 primers: forward 5’-CTCTTCCACGGCAACCAAAA-3’, reverse 5’-AGGGGCCATCCACAGTCTTC-3’.

The article "Repressing phosphatidylinositol-4,5-bisphosphate 3-kinase catalytic subunit gamma by microRNA-142-3p restrains the progression of hepatocellular carcinoma" was retracted in 2024. Reasons: original data or images not available; unreliable results or conclusions; concerns about the data; concerns about the results or conclusions.

### Western blot (WB)

After cell treatment, the medium was discarded. Supplementation of protein lysis solution (Roche) was completed for separating the total protein. Then, 50 μg of total protein was sampled on 12% polyacrylamide gel for 2-hour electrophoresis at 100 V. Afterward, the electrophoresed total protein was transferred to polyvinylidene fluoride (PVDF) membranes. One hour after being sealed with 5% skimmed milk at RT, the membranes were flushed three times (10 minutes each time) with Tris-buffered saline with Tween-20 (TBST) for overnight incubation at 4°C with the following primary antibodies (Abcam, Cambridge, UK, concentration 1:1000): Anti-Bax antibody (ab182734), Anti-Bcl-2 antibody (ab692), Anti-Cleaved Caspase-3 antibody (ab214430), Anti-p-AKT antibody (ab38449), Anti-AKT antibody (ab8805), Anti-p-PI3K antibody (ab278545), Anti-PI3K antibody (ab140307), and Anti-HIF-1 alpha Antibody (ab179483). Next, the membranes were maintained with the horseradish peroxidase (HRP)-labeled Goat Anti-Rabbit IgG (ab6205718) (concentration 1:2500) at RT for one hour after being rinsed with TBST. Following 3 washes with TBST (10 minutes/time), the membranes were exposed with enhanced chemiluminescence (ECL) chromogenic agent (Millipore, Bedford, MA, USA), and a membrane scanner was utilized for imaging [24].

### The dual-luciferase reporter assay

The wild-type (WT) and mutant-type (MUT) sequences of the PIK3CG-3’-untranslated region (UTR) were synthesized by GenePharma (Shanghai, China) and inserted into the pmiR-GLO dual-luciferase vector. WT PIK3CG-3’-UTR and MUT PIK3CG-3’-UTR were employed to transfect 293 T cells that overexpressed miR-142-3p or its control with Lipofectamine 2000 (Invitrogen, USA). Renilla luciferase expression plasmids were transfected into cells as an endogenous control. Forty-eight hours later, we lysed the harvested cells with a lysis buffer (Promega, USA). Firefly and renilla luciferase activities were examined by the Dual-Luciferase Reporter Assay System (Promega, USA), following the manufacturer’s instructions [25].

### RNA immunoprecipitation (RIP)

To probe the interrelationship between miR-142-3p and PIK3CG, RIP was completed adopting the Magna RIP™ RNA-binding protein immunoprecipitation kit (Millipore, Bedford, MA, USA). The transfection of Huh-7 cells (2 × 10^7^) was carried out with miR-142-3p mimics or miR-NC. Next, the cells were obtained to be affiliated with 200 µL of RIP Lysis Buffer. Five minutes after being lysed on ice, the cells underwent 15-minute centrifugation at 1500 rpm for the acquirement of the supernatant. Afterward, the anti-Argonaute 2 (Ago2) or anti-IgG (Sigma) was adopted for overnight incubation of the extract. After 5 washes of the magnetic beads with the washing buffer solution, the supernatant was removed. Protease K lysate was then added to magnetic beads and lysed at 55°C for 30 minutes. In the end, the supernatant was transferred to a fresh centrifuge tube. Phenol–chloroform-isoamyl alcohol was employed for extracting the total RNA. For the purification, isopropanol centrifugation was adopted. The co-precipitated RNA was separated and analyzed by qRT-PCR to verify the existence of the binding targets [20].

The article "Repressing phosphatidylinositol-4,5-bisphosphate 3-kinase catalytic subunit gamma by microRNA-142-3p restrains the progression of hepatocellular carcinoma" was retracted in 2024. Reasons: original data or images not available; unreliable results or conclusions; concerns about the data; concerns about the results or conclusions.

### Immunohistochemistry (IHC)

HCC tissues and matched non-tumor tissues were immobilized in 4% formalin and paraffin-embedded. After blocking, the tissues were sliced into 4-μM sections for overnight incubation with the primary antibodies of the Anti-AKT antibody (ab8805), Anti-PI3K antibody (ab140307), Anti-HIF-1 alpha antibody (ab179483), and Anti-PIK3CG antibody (ab277879) (Biorbyt, Cambridge, UK) at 4°C. After being rinsed with PBS, the sections underwent 1-hour incubation with the secondary antibody at 37°C for the 3-minute staining with the 3,3-diaminobenzidine solution. Finally, nuclei counterstaining was performed with hematoxylin [26].

### TdT-mediated dUTP nick end labeling (TUNEL) staining

For the assessment of cell apoptosis *in vivo*, all specimens were subject to overnight fastening in 4% paraformaldehyde at 4°C. Next, 0.1% Triton X-100 was adopted for permeabilization. Under the manufacturer’s instruction, the 1-hour incubation of the specimens was carried out with the TUNEL staining solution (Beyotime, Haimen, China). The microscope (Olympus) was employed for counting TUNEL-positive cells in five randomly selected fields of the slides [25].

### Fluorescence in situ hybridization (FISH)

HCC tissues were immobilized in 4% paraformaldehyde, dehydrated in 70%, 95% and 100% ethanol and hybridized overnight at 37°C in a dark humid chamber. After hybridization, slides were flushed thrice in 60 mL of 50% formamide/2X SSC and left to incubate overnight at 4°C with miR-142-3p-labeled probe. Following three washes at RT, the slides were maintained with TSA Fluorescence Signal Response Solution (PerkinElmer, NEL701001KT, TSA Fluorescein system) for 30 minutes and sealed with a DAPI-containing tablet. Images were captured with a fluorescent microscope (Leica, SP8 laser confocal microscopy) to allow the assessment of miR-142-3p expression levels in liver cancer tissues.

The article "Repressing phosphatidylinositol-4,5-bisphosphate 3-kinase catalytic subunit gamma by microRNA-142-3p restrains the progression of hepatocellular carcinoma" was retracted in 2024. Reasons: original data or images not available; unreliable results or conclusions; concerns about the data; concerns about the results or conclusions.

### Tumor formation experiment in nude mice

For the establishment of an *in-vivo* tumor formation model, 6-week-old BALB/c-nu nude mice (ordered from the Animal Center of Zhejiang University) were utilized. Subsequently, 0.25% trypsin was employed for trypsinizing Huh7 cells in the logarithmic growth phase. The cells were harvested, rinsed, and resuspended with the serum-free medium to make single-cell suspensions (3 × 10^8^/mL). Each mouse was subcutaneously administered with 0.1 mL of cell suspension into the axilla of the left forelimb. A total of 20 mice were used, with 10 mice in each group. After the administration, the mice were anesthetized on days 7, 14, 21, 28 and 35 for removing the tumors and measuring tumor weights. The longest diameter of the tumor (a) and its perpendicular shortest diameter (b) were gauged with a vernier caliper. The tumor volume was calculated as per the following formula: V(mm^3^) = 0.5 × a × b [2]. All experiments met the authorization of the Animal Experiment Ethics Review Committee of HuaMei Hospital of University of Chinese Academy of Science. The experiment was implemented strictly under the National Institutes of Health Laboratory Animal Care and Use Guidelines (NIH Publication No. 8023) [27].

## Statistical analysis

The analysis was made with the SPSS 24.0 statistical software (IBM Corp., Armonk, NY, USA). Measurements were represented as mean ± variance (x ± s). *t* test was implemented for comparison between the two groups, and analysis of variance was adopted for comparing the mean difference between groups. The enumeration data were represented by fourfold tables (or percentages), and the difference between the two groups was analyzed by applying χ2 test. The difference had statistical meaning when *P*< 0.05. [22]

## Results

### miR-142-3p expression is lowered in HCC tissues and cell lines

To elucidate the expression characteristics of miR-142-3p in HCC tissues and cell lines, we examined the miR-142-3p profile in HCC tissues and paracancerous non-tumor tissues as well as in HCC cells and normal hepatocytes. Also, we queried the Starbase database for miR-142-3p profiles in HCC and conducted a correlation analysis between miR-142-3p expression and clinicopathological features of HCC patients. As indicated by qRT-PCR, by contrast with that in adjacent healthy tissues, miR-142-3p presented marked down-regulation in HCC tissues (*P*< 0.05, Figure 1a). FISH checked the localization of miR-142-3p in HCC tissues and non-tumor liver tissues. It was revealed that miR-142-3p was mainly expressed in the cytoplasm of non-tumor tissues and was less expressed in HCC tissues (Figure 1b). In the Starbase database (http://starbase.sysu.edu.cn/), miR-142-3p also had lower levels in HCC tissues (Figure 1c). Furthermore, by contrast with that in human normal liver cell L-O2, miR-142-3p expression was dramatically diminished in HCC cell lines (HCCLM3 and Huh-7) (*P*< 0.05, Figure 1d). More importantly, HCC patients with low miR-142-3p expression had larger tumor volume and later tumor stage and were more likely to have vascular infiltration (Table 1). Additionally, HCC patients with high miR-142-3p expression had longer survival periods than those with low miR-142-3p expression (Figure 1e), which was also affirmed by the Starbase (Figure 1f). Thus, miR-142-3p was downregulated in HCC.

The article "Repressing phosphatidylinositol-4,5-bisphosphate 3-kinase catalytic subunit gamma by microRNA-142-3p restrains the progression of hepatocellular carcinoma" was retracted in 2024. Reasons: original data or images not available; unreliable results or conclusions; concerns about the data; concerns about the results or conclusions.

**Table 1.** Interrelationship between miR-142-3p expression and clinical characters in tissue specimens of HCC patients

Characteristics	Patients	Expression of miR-142-3p	P-value	
	High-miR-142-3p		Low-miR-142-3p	
Total	50	19	31	
Age(years)				
<60	15	7	8	0.408
≥60	35	12	23	
Gender				
Male	37	16	21	0.198
Female	13	3	10	
Tumor size				
<5	29	15	14	0.019*
≥5	21	4	17	
Serum AFP (ng/ml)				
<20	14	8	6	0.082
≥20	36	11	25	
Liver cirrhosis				
Absent	7	4	3	0.261
Presen		43	15	28
Vascular invasion				
NO	33	16	17	0.033*
Yes	17	3	14	
Edmondson grade				
I–II	30	15	15	0.032*
III–IV	20	4	16	
Tumor multiplicity				
Single	35	14	21	0.656
Multiple	15	5	10	

(Note: *P< 0.05 has statistical significance)

**Figure 1.** **miR-142-3p presents a diminution in HCC tissues and cell lines**. A: miR-142-3p expression was gauged in HCC tissues and adjacent healthy tissues by qRT-PCR. B: Localization of miR-142-3p in HCC tissues and non-tumor liver tissues was monitored by FISH assay. C. The expression characteristics of miR-142-3p in HCC tissues and adjacent non-tumor tissues were verified via the Starbase database. D: qRT-PCR assayed miR-142-3p levels in liver cells and HCC cell lines. E: Prognostic analysis of miR-142-3p in HCC. F. Overall survival of HCC patients with high and low expression of miR-142-3p. ***P< 0.001 (vs. Normal group). ***P< 0.001 (vs. L-O2 group).

### miR-142-3p overexpression dampens proliferation and accelerates apoptosis of HCC cells

To inquire into the biological impact of miR-142-3p overexpression on HCC cells, miR-NC and miR-142-3p mimics were transfected into HCC cells (Huh7 and HCCLM3). The transfection validity was assessed 48 hours later with qRT-PCR, which corroborated that miR-142-3p was distinctly up-regulated in HCC cells transfected with miR-142-3p mimics versus the miR-NC group (*P*< 0.05, Figure 2a). Cell proliferation was gauged by applying the colony formation assay and BrdU staining. As a result, overexpressing miR-142-3p prominently dampened Huh7 and HCCLM3 cell proliferation versus the control group (*P*< 0.05, Figure 2b-c). Additionally, the FCM data exhibited that transfecting miR-142-3p mimics facilitated Huh7 and HCCLM3 cell apoptosis versus the control group (*P*< 0.05, Figure 2d). Moreover, the Transwell assay disclosed that Huh7 and HCCLM3 cell migration and invasion exhibited considerable inhibition after transfecting miR-142-3p mimics versus the control group (*P*< 0.05, Figure 2e-f). The expression of apoptosis-related proteins was further assayed by WB. It turned out that the expression of pro-apoptotic proteins Bax and Cleaved-caspase3 was notably raised, and the expression of anti-apoptotic protein Bcl2 showed a noticeable decline in the miR-142-3p overexpression group (vs. the control group) *(P *< 0.05, Figure 2g). These outcomes validated that transfecting miR-142-3p mimics in Huh7 and HCCLM3 cells impeded the tumorigenic phenotype of HCC cells.

The article "Repressing phosphatidylinositol-4,5-bisphosphate 3-kinase catalytic subunit gamma by microRNA-142-3p restrains the progression of hepatocellular carcinoma" was retracted in 2024. Reasons: original data or images not available; unreliable results or conclusions; concerns about the data; concerns about the results or conclusions.

**Figure 2.** **Overexpressing miR-142-3p restrains HCC cell proliferation and facilitates cell apoptosis**. The transfection of miR-142-3p mimics was carried out in Huh7 and HCCLM3 cells. A: For the measurement of miR-142-3p expression in Huh7 and HCCLM3, qRT-PCR was carried out. B-C: The colony formation assay and BrdU staining were applied for the examination of cell proliferation. D: For the detection of cell apoptosis, FCM was performed. E-F: The migration and invasion of Huh7 and HCCLM3 cells were assayed by the Transwell experiment. G: WB tested the expression of Bax, Bcl2 and Cleaved-caspase3. *P< 0.05, **P< 0.001 (vs. miR-NC group) N = 3.

### Knocking down miR-142-3p causes the acceleration of HCC cell proliferation and represses apoptosis

To ascertain the impact of miR-142-3p on HCC, miR-in and miR-142-3p inhibitors were transfected into HCC cells (Huh7 and HCCLM3). Transfection efficiency was monitored after 48 hours with qRT-PCR, which displayed that miR-142-3p was down-regulated in HCC cells transfected with miR-142-3p inhibitors versus the miR-in group (*P*< 0.05, Figure 3a). Cell proliferation was checked by employing the colony formation assay and BrdU staining. The outcomes suggested that knocking down miR-142-3p caused an outstanding acceleration of proliferation in Huh7 and HCCLM3 cells (vs. the control group) (*P*< 0.05, Figure 3b-c). Besides, FCM data exhibited that transfecting miR-142-3p inhibitors restrained Huh7 and HCCLM3 cell apoptosis (vs. the control group) (*P*< 0.05, Figure 3d). Moreover, the Transwell assay unveiled that by contrast with the control group, the migration and invasion of Huh7 and HCCLM3 cells presented substantial elevation after transfecting miR-142-3p inhibitors (*P*< 0.05, Figure 3e-f). The expression of apoptosis-related proteins was further assayed by WB. It turned out that the expression of Bax and Cleaved-caspase3 in the miR-142-3p knockdown group was declined, whereas the expression of Bcl2 presented prominent up-regulation (vs. the control group) (*P*< 0.05, Figure 3g). The above evidence implied that transfecting miR-142-3p inhibitors in Huh7 and HCCLM3 cells expedited the malignant phenotype of HCC cells.

The article "Repressing phosphatidylinositol-4,5-bisphosphate 3-kinase catalytic subunit gamma by microRNA-142-3p restrains the progression of hepatocellular carcinoma" was retracted in 2024. Reasons: original data or images not available; unreliable results or conclusions; concerns about the data; concerns about the results or conclusions.

**Figure 3.** **Knocking down miR-142-3p accelerates HCC cell proliferation and dampens cell apoptosis**. miR-142-3p inhibitors were transfected into Huh7 and HCCLM3. A: miR-142-3p expression in Huh7 and HCCLM3 HCC cells was gauged by qRT-PCR. B-C: Cell proliferation was checked by employing the colony formation assay and BrdU staining. D: FCM measured cell apoptosis. E-F: The Transwell experiment assayed the migration and invasion of Huh7 and HCCLM3 cells. G: WB evaluated the expression of the apoptosis-related proteins. *P< 0.05, **P< 0.01,***P< 0.001, ****P< 0.0001 (vs. miR-NC group) N = 3.

### Knockdown of miR-142-3p facilitates HCC cell development in vivo

We have explored the biological effects of miR-142-3p on HCC cells in an *in-vitro* model. Next, we injected Huh7 cells transfected with miR-in and miR-142-3p inhibitors into the nude mice to establish an *in-vivo* tumorigenic model to further validate the influence of knocking down miR-142-3p on HCC cell growth and apoptosis *in vivo*. As a result, knocking down miR-142-3p brought about the promotion of tumor size and weight (*P*< 0.05, Figure 4a-c). WB findings manifested that the expression of Bax and Cleaved-caspase3 presented a diminution after knocking down miR-142-3p, while the expression of anti-apoptotic protein Bcl2 was lifted (vs. the miR-in group) (*P*< 0.05, Figure 4d). The findings of the TUNEL experiment manifested that the TUNEL-positive cell number was markedly reduced after suppressing miR-142-3p (*P*< 0.05, Figure 4e). These discoveries implied that restraining miR-142-3p expedited HCC cell development *in vivo*.

**Figure 4.** **Knocking down miR-142-3p accelerates HCC development *in vivo.*** A: Tumor growth map in nude mice. B-C: After 35 days, the mice were killed, the subcutaneous tumors were harvested, and the tumor volume and weight were gauged. D: WB measured the expression of the apoptosis-related proteins after restraining miR-142-3p expression *in vivo*. E: The TUNEL experiment assayed tumor cell apoptosis. ns*P*>0.05, *P< 0.05, **P< 0.01, ***P< 0.001, ****P< 0.0001 (vs. miR-in group). N = 5.

### The influence of inhibiting miR-142-3p on the PI3K/AKT/HIF-1α axis

To delve into the specific molecular mechanism of miR-142-3p in HCC evolution, we checked the PI3K/AKT/HIF-1α pathway profile both *in vivo* and *in vitro* and tested the positive expression of the PI3K/AKT/HIF-1α pathway in HCC tissues. As testified by WB, the pathway expression in the miR-142-3p-in group exhibited remarkable up-regulation versus the miR-in group *in vivo* (*P*< 0.05, Figure 5a). Meanwhile, IHC further assayed the positive expression of the pathway in HCC cancer tissues. The results illuminated that the positive cell number of the PI3K/AKT/HIF-1α pathway was augmented after suppressing miR-142-3p (vs. the miR-in group) (*P*< 0.05, Figure 5b). *In vitro*, overexpressing miR-142-3p restrained the PI3K/AKT/HIF-1α pathway expression, while knocking down miR-142-3p exerted the reverse effect (Figure 5c, d). These outcomes signified that miR-142-3p knockdown facilitated the PI3K/AKT/HIF-1α pathway activation.

The article "Repressing phosphatidylinositol-4,5-bisphosphate 3-kinase catalytic subunit gamma by microRNA-142-3p restrains the progression of hepatocellular carcinoma" was retracted in 2024. Reasons: original data or images not available; unreliable results or conclusions; concerns about the data; concerns about the results or conclusions.

**Figure 5.** **The influence of inhibiting miR-142-3p on the PI3K/AKT/HIF-1α axis**. The miR-142-3p knockdown model was constructed in Huh7 cells. A: WB examined the PI3K/AKT/HIF-1α pathway expression. B: IHC assayed the positive expression of PI3K/AKT/HIF-1α in HCC tissues. C-D: WB examined the PI3K/AKT/HIF-1α pathway expression in miR-142-3p overexpression and knockdown HCC cell models. **P< 0.01, ***P< 0.001, ****P< 0.0001 (vs. miR-in group). N = 3.

### miR-142-3p targets PIK3CG

By checking the Starbase database, we determined that PIK3CG is a possible target for miR-142-3p. To define the targeting association of miR-142-3p with PIK3CG, we implemented a dual-luciferase reporter assay and a RIP assay. Additionally, we assayed PIK3CG profiles in a miR-142-3p knockdown cell model and tested the number of PIK3CG-positive cells in HCC tissues. The Starbase database identified a possible targeting link between miR-142-3p and PIK3CG (Figure 6a). In parallel, the dual-luciferase reporter assay outcomes uncovered that miR-142-3p restrained the PIK3CG-WT activity (*P*< 0.05, Figure 6b), while it had no noticeable impact on PIK3CG-MUT (*P*> 0.05, Figure 6b). Furthermore, the RIP data exhibited that the amount of PIK3CG precipitated in the Ago2 antibody group was higher than that in the IgG group after the transfection of miR-142-3p, suggesting that PIK3CG bound with Ago2 via miR-142-3p (*P*< 0.05, Figure 6c). Next, we monitored the PIK3CG expression after miR-142-3p knockdown in Huh7 cells. Compared with the miR-in group, knocking down miR-142-3p facilitated PIK3CG expression (*P*< 0.05, Figure 6d). IHC unveiled that miR-142-3p knockdown markedly heightened the PIK3CG-positive cell number versus the miR-in group (*P*< 0.05, Figure 6e). Hence, miR-142-3p targeted and reversely regulated PIK3CG expression in HCC cells.

The article "Repressing phosphatidylinositol-4,5-bisphosphate 3-kinase catalytic subunit gamma by microRNA-142-3p restrains the progression of hepatocellular carcinoma" was retracted in 2024. Reasons: original data or images not available; unreliable results or conclusions; concerns about the data; concerns about the results or conclusions.

**Figure 6.** **miR-142-3p is targeted by PIK3CG**. A: The Starbase database predicted the binding target between PIK3CG and miR-142-3p. B: The relative luciferase activity was assayed 48 hours after transfection of 293 T cells with miR-142-3p mimics or NC mimics and PIK3CG-WT or PIK3CG-MT. C: RIP validated the exact interaction between PIK3CG and miR-142-3p. D: qRT-PCR tested PIK3CG expression in Huh7 cells. E: PIK3CG-positive cells in living tumor tissues was monitored by IHC. ns*P*>0.05, ***P< 0.001. N = 3.

### PIK3CG overexpression attenuates the anti-tumor effect of miR-142-3p in HCC cells

To make certain the impact of PIK3CG on the anti-tumor effect of miR-142-3p in HCC progression, we transfected miR-NC, miR-142-3p mimics and miR-142-3p mimics + PIK3CG overexpression plasmids into HCCLM3 cells and then gauged cell proliferation, apoptosis, migration, and invasion and the PI3K/AKT/HIF-1α pathway expression. The qRT-RCR assay displayed that miR-142-3p overexpression retarded the PIK3CG expression versus the miR-NC group. In contrast, PIK3CG was notably up-regulated in HCC cells in the miR-142-3p + PIK3CG group versus the miR-142-3p group (*P*< 0.05, Figure 7a). The colony formation assay and BrdU staining were adopted for evaluating cell proliferation. It was presented that compared with the miR-142-3p group, PIK3CG overexpression accelerated HCCLM3 cell proliferation (*P*< 0.05, Figure 7b-c). Furthermore, FCM findings substantiated that HCCLM3 cell apoptosis in the miR-142-3p+PIK3CG group exhibited a reduction (vs. the miR-142-3p group) (*P*< 0.05, Figure 7d). Transwell assay illuminated that in comparison to the miR-142-3p group, HCCLM3 cell migration and invasion were augmented in the miR-142-3p+PIK3CG group (*P*< 0.05, Figure 7e). The profiles of apoptosis-related proteins were further tested by WB. It turned out that Bax and Cleaved-caspase3 expression presented an appreciable decline, while Bcl2 was up-regulated in the miR-142-3p+PIK3CG group (vs. the miR-142-3p group) (*P*< 0.05, Figure 7f). Meanwhile, compared to the miR-142-3p group, the PI3K/AKT/HIF-1α pathway profile was elevated in the miR-142-3p+PIK3CG group (*P*< 0.05, Figure 7g). Thus, overexpressing PIK3CG attenuated the tumor-suppressive effect of miR-142-3p in HCC and accelerated HCC development.

**Figure 7.** **Overexpressing PIK3CG weakens the anti-tumor effects of miR-142-3p in HCC cells**. The miR-NC, miR-142-3p mimic, and miR-142-3p mimic + PIK3CG overexpression plasmids were transfected into HCCLM3 cells. A: qRT-PCR examined PIK3CG expression. B-C: The colony formation assay and BrdU staining were conducted for the measurement of cell proliferation. D: FCM assayed cell apoptosis. E: Migration and invasion of HCCLM3 cells were gauged by the Transwell experiment. F-G: WB assayed the expression of the apoptosis-related proteins and PI3K/AKT/HIF-1α. **P< 0.01, ***P< 0.001, ****P< 0.0001 (vs. miR-NC group). &*P*< 0.05, &&*P*< 0.05, &&&*P*< 0.001 (vs. miR-142-3p group). N = 3.

The article "Repressing phosphatidylinositol-4,5-bisphosphate 3-kinase catalytic subunit gamma by microRNA-142-3p restrains the progression of hepatocellular carcinoma" was retracted in 2024. Reasons: original data or images not available; unreliable results or conclusions; concerns about the data; concerns about the results or conclusions.

## Discussion

MiRNAs, which exert pivotal properties in molecular functions and pathological significance in HCC [28,29], are promising therapeutic targets for HCC diagnosis and prognosis. This paper has unveiled that miR-142-3p expression exhibits a reduction in HCC tissues and cell lines. Meanwhile, miR-142-3p dampens HCC cells’ proliferation, migration and invasion and facilitates their apoptosis by acting as a tumor suppressor. Besides, the study has initially elucidated that miR-142-3p targets the 3’-UTR of PIK3CG and impedes the HCC progression by targeting PIK3CG. These discoveries manifest that miR-142-3p exerts vital parts in HCC and may become a novel therapeutic target for HCC.

As a tumor suppressor, miR-142-3p is dysregulated in diverse cancers. For instance, miR-142-3p exhibits an outstanding decline in non-small cell lung cancer (NSCLC). Overexpressing miR-142-3p remarkably chokes NSCLC cell proliferation, migration, and invasion [30]. Furthermore, miR-142-3p is markedly diminished in lung adenocarcinoma tissues and cell lines. Overexpressing miR-142-3p negatively modulates nuclear receptor subfamily 2 group F member 6 (NR2F6) to restrain cell proliferation, migration and invasion and facilitate cell apoptosis *in vitro* [31]. Consistent with the above studies, we observe that miR-142-3p shows a reduction in HCC tissues and cell lines. Overexpressing miR-142-3p restrains the malignant behaviors of HCC cells. Nevertheless, the inverse results are obtained following the miR-142-3p knockdown, which is testified *in vivo*. These findings further validate the anti-tumor effect of miR-142-3p in HCC, offering a crucial reference for the molecular targeting therapy of HCC.

Previous reports have elucidated that these miRNAs facilitate mRNA degradation or restrain mRNA translation to modulate gene expression, thereby controlling the proliferation, differentiation, apoptosis, invasion, migration and angiogenesis of cancer cells [32]. The modulation of miR-142-3p on mRNAs influences the development of various tumors. miR-142-3p has been claimed to restrain cervical cancer cell proliferation by negatively modulating HMGB1 [33]. Furthermore, the β-catenin gene (CTNNB1) is directly targeted by miR-142-3p, which chokes the Wnt signal and thus exerts its tumor-suppressive effects in colorectal cancer [34]. In addition, Li Z et al. reveal that miR-142-3p suppresses the malignant progression of endometrial cancer by targeting and negatively regulating the family with sequence similarity 98 member A (FAM98A) [35]. To figure out the mechanism of miR-142-3p’s effect on HCC cell biology, we employed a bioinformatics website for predicting miR-142-3p’s potential target. The database exhibited that PIK3CG was the direct target of miR-142-3p, which was testified by the dual-luciferase reporter assay and RIP experiment. The rescue experiment exhibited that PIK3CG overexpression weakened the suppressive effect of miR-142-3p on HCC cell proliferation and migration. These outcomes hinted that PIK3CG restrained the anti-tumor properties of miR-142-3p.

The article "Repressing phosphatidylinositol-4,5-bisphosphate 3-kinase catalytic subunit gamma by microRNA-142-3p restrains the progression of hepatocellular carcinoma" was retracted in 2024. Reasons: original data or images not available; unreliable results or conclusions; concerns about the data; concerns about the results or conclusions.

The dysregulation of the signal has an association with cancers. As reported, the aberrant expression of the PI3K/AKT/HIF-1α axis has involvement in the biological processes of numerous tumors. Chen J et al. have reported that Gankyrin expedites the proliferation of ovarian cancer cells driven by follicle-stimulating hormone via the PI3K/AKT/HIF-1α/cyclin D1 pathway activation [36]. Gao L et al. have illustrated that CD90 stimulates the PI3K/AKT/HIF-1α pathway to intensify the malignant biological behaviors of gastric cancer (GC), disrupting energy metabolism [37]. Besides, inhibiting the PI3K/AKT/HIF-1α pathway improves the therapeutic effect of paclitaxel in GC [38]. Meanwhile, activating the pathway favors the hypoxia-induced EMT and chemoresistance of HCC cells, thus aggravating the malignant progression of HCC [39]. These data have manifested that activating the PI3K/AKT/HIF-1α signal boosts malignant behaviors of various malignancies, and blocking this pathway is expected to be an underlying strategy to treat tumors. Fortunately, in agreement with the above research, our IHC findings revealed that knocking down miR-142-3p lessened the number of PI3K/AKT/HIF-1α-positive cells. Cell experiment results elucidated that knocking down miR-142-3p markedly dampened the PI3K/AKT/HIF-1α expression, restrained HCC cell proliferation, migration and invasion and facilitated cell apoptosis. Hence, miR-142-3p hampered HCC progression by dampening the PI3K/AKT/HIF-1α axis.

## Conclusion

In summary, our research manifests that miR-142-3p is down-regulated in HCC tissues and cells. Overexpressing miR-142-3p restrains HCC cells’ proliferation, migration and invasion *in vitro*, and knocking down miR-142- 3p expedites the growth and metastasis of xenograft tumors *in vivo*. Additionally, miR-142-3p suppressed the PI3K/AKT/HIF-1α signaling activity by binding to the 3’-UTR of PIK3CG to impede PIK3CG expression. This research provides valuable clues for developing new therapeutic targets for HCC. However, more molecular mechanisms require to be further probed.

The article "Repressing phosphatidylinositol-4,5-bisphosphate 3-kinase catalytic subunit gamma by microRNA-142-3p restrains the progression of hepatocellular carcinoma" was retracted in 2024. Reasons: original data or images not available; unreliable results or conclusions; concerns about the data; concerns about the results or conclusions.

## Data Availability

The data sets used and analyzed during the current study are available from the corresponding author on reasonable request.

## References

[1] Wallace MC, Preen D, Jeffrey GP, et al. The evolving epidemiology of hepatocellular carcinoma: a global perspective. Expert Rev Gastroenterol Hepatol. 2015 Jun;9(6):765–779.2582782110.1586/17474124.2015.1028363

[2] Feng RM, Zong YN, Cao SM, et al. Current cancer situation in China: good or bad news from the 2018 Global Cancer Statistics? Cancer Commun (Lond). 2019 Apr 29;39(1):22.3103066710.1186/s40880-019-0368-6PMC6487510

[3] Zheng J, Zhu MY, Wu F, et al. A blood-based 22-gene expression signature for hepatocellular carcinoma identification. Ann Transl Med. 2020 Mar;8(5):195.3230934210.21037/atm.2020.01.93PMC7154425

[4] Zhang X, Li J, Shen F, et al. Significance of presence of microvascular invasion in specimens obtained after surgical treatment of hepatocellular carcinoma. J Gastroenterol Hepatol. 2018 Feb;33(2):347–354.2858963910.1111/jgh.13843

[5] Chen L, Heikkinen L, Wang C, et al. Trends in the development of miRNA bioinformatics tools. Brief Bioinform. 2019 Sep 27;20(5):1836–1852.2998233210.1093/bib/bby054PMC7414524

[6] Lyu P, Zhai Z, Hao Z, et al. CircWHSC1 serves as an oncogene to promote hepatocellular carcinoma progression. Eur J Clin Invest. 2021 Jan;6:e13487.10.1111/eci.1348733410156

[7] Cui D, Ni C. LncRNA Lnc712 promotes tumorigenesis in hepatocellular carcinoma by targeting miR-142-3p/Bach-1 Axis. Cancer Manag Res. 2020 Nov 5;12: 11285–11294.3317787810.2147/CMAR.S254950PMC7652235

[8] Yu Q, Xiang L, Chen Z, et al. MALAT1 functions as a competing endogenous RNA to regulate SMAD5 expression by acting as a sponge for miR-142-3p in hepatocellular carcinoma. Cell Biosci. 2019 May 10;9(1):39.3116835510.1186/s13578-019-0299-6PMC6509837

[9] Fu Y, Sun LQ, Huang Y, et al. miR-142-3p Inhibits the Metastasis of Hepatocellular Carcinoma Cells by Regulating HMGB1 Gene Expression. Curr Mol Med. 2018;18(3):135–141.3019843210.2174/1566524018666180907161124

[10] Liu J, Huang B, Xiu Z, et al. PI3K/Akt/HIF-1α signaling pathway mediates HPV-16 oncoprotein-induced expression of EMT-related transcription factors in non-small cell lung cancer cells. J Cancer. 2018 Sep 8;9(19):3456–3466.3031050210.7150/jca.26112PMC6171031

[11] Zhou J, Schmid T, Frank R, et al. PI3K/Akt is required for heat shock proteins to protect hypoxia-inducible factor 1alpha from pVHL-independent degradation. J Biol Chem. 2004 Apr 2;279(14):13506–13513.1472652910.1074/jbc.M310164200

The article "Repressing phosphatidylinositol-4,5-bisphosphate 3-kinase catalytic subunit gamma by microRNA-142-3p restrains the progression of hepatocellular carcinoma" was retracted in 2024. Reasons: original data or images not available; unreliable results or conclusions; concerns about the data; concerns about the results or conclusions.

[12] Yun SP, Lee MY, Ryu JM, et al. Role of HIF-1alpha and VEGF in human mesenchymal stem cell proliferation by 17beta-estradiol: involvement of PKC, PI3K/Akt, and MAPKs. Am J Physiol Cell Physiol. 2009 Feb;296(2):C317–26.1898724910.1152/ajpcell.00415.2008

[13] Liu X, Liu L, Chen K, et al. Huaier shows anti-cancer activities by inhibition of cell growth, migration and energy metabolism in lung cancer through PI3K/AKT/HIF-1α pathway. J Cell Mol Med. 2021 Feb;25(4):2228–2237.3337761910.1111/jcmm.16215PMC7882940

[14] Liao ZH, Zhu HQ, Chen YY, et al. The epigallocatechin gallate derivative Y6 inhibits human hepatocellular carcinoma by inhibiting angiogenesis in MAPK/ERK1/2 and PI3K/AKT/ HIF-1α/VEGF dependent pathways. J Ethnopharmacol. 2020;259:112852.3227875910.1016/j.jep.2020.112852

[15] Yu L, Sun Y, Li J, et al. Silencing the Girdin gene enhances radio-sensitivity of hepatocellular carcinoma via suppression of glycolytic metabolism. J Exp Clin Cancer Res. 2017 Aug 15;36(1):110.2881089610.1186/s13046-017-0580-7PMC5558715

[16] Chung WC, Zhou X, Atfi A, et al. PIK3CG is a potential therapeutic target in androgen receptor-indifferent metastatic prostate cancer. Am J Pathol. 2020 Nov;190(11):2194–2202.3280523410.1016/j.ajpath.2020.07.013

[17] Wang J, Li M, Han X, et al. MiR-1976 knockdown promotes epithelial-mesenchymal transition and cancer stem cell properties inducing triple-negative breast cancer metastasis. Cell Death Dis. 2020 Jul 3;11(7):500.3262074810.1038/s41419-020-2711-xPMC7335055

[18] Chen S, Li F, Chai H, et al. miR-502 inhibits cell proliferation and tumor growth in hepatocellular carcinoma through suppressing phosphoinositide 3-kinase catalytic subunit gamma. Biochem Biophys Res Commun. 2015 Aug 21;464(2):500–505.2616326410.1016/j.bbrc.2015.06.168

[19] Zhang R, Guo C, Liu T, et al. MicroRNA miR-495 regulates the development of Hepatocellular Carcinoma by targeting C1q/tumor necrosis factor-related protein-3 (CTRP3). Bioengineered. 2021 Dec;12(1):6902–6912. PMID: 34516334.3451633410.1080/21655979.2021.1973878PMC8806502

[20] Zheng S, Guo Y, Dai L, et al. Long intergenic noncoding RNA01134 accelerates hepatocellular carcinoma progression by sponging microRNA-4784 and downregulating structure specific recognition protein 1. Bioengineered. 2020 Dec;11(1):1016–1026. PMID: 32970959.3297095910.1080/21655979.2020.1818508PMC8291876

[21] Fu C, Li J, Li P, et al. LncRNA DNAJC3-AS1 Promotes Hepatocellular Carcinoma (HCC) progression via sponging premature miR-27b. Cancer Manag Res. 2021 Nov15;13:8575–8583. PMID: 34815712.3481571210.2147/CMAR.S321111PMC8604638

[22] Zhou X, Chang Y, Zhu L, et al. LINC00839/miR-144-3p/WTAP (WT1 Associated Protein) axis is involved in regulating hepatocellular carcinoma progression. Bioengineered. 2021 Oct 11. Epub ahead of print. PMID: 34634995. DOI:10.1080/21655979.2021.1990578PMC880996934634995

The article "Repressing phosphatidylinositol-4,5-bisphosphate 3-kinase catalytic subunit gamma by microRNA-142-3p restrains the progression of hepatocellular carcinoma" was retracted in 2024. Reasons: original data or images not available; unreliable results or conclusions; concerns about the data; concerns about the results or conclusions.

[23] Zhu X, Jiang S, Wu Z, et al. Long non-coding RNA TTN antisense RNA 1 facilitates hepatocellular carcinoma progression via regulating miR-139-5p/SPOCK1 axis. Bioengineered. 2021 Dec;12(1):578–588. PMID: 33517826.3351782610.1080/21655979.2021.1882133PMC8291788

[24] Zhou Y, Li K, Zou X, et al. LncRNA DHRS4-AS1 ameliorates hepatocellular carcinoma by suppressing proliferation and promoting apoptosis via miR-522-3p/SOCS5 axis. Bioengineered. 2021 Oct 20. Epub ahead of print. PMID: 34666613. 10.1080/21655979.2021.1994719PMC880996334666613

[25] Li Y, Jiang A. ST8SIA6-AS1 promotes hepatocellular carcinoma by absorbing miR-5195-3p to regulate HOXB6. Cancer Biol Ther. 2020Jul2;21(7):647–655. Epub 2020 May 18. PMID: 32420798.3242079810.1080/15384047.2020.1743150PMC7515456

[26] Wang J, He H, Jiang Q, et al. CBX6 Promotes HCC metastasis via transcription factors Snail/Zeb1-Mediated EMT mechanism. Onco Targets Ther. 2020 Dec4;13:12489–12500. PMID: 33311989.3331198910.2147/OTT.S257363PMC7727033

[27] Li M, Shao J, Guo Z, et al. Novel mitochondrion-targeting copper(II) complex induces HK2 malfunction and inhibits glycolysis via Drp1-mediating mitophagy in HCC. J Cell Mol Med. 2020 Mar;24(5):3091–3107. Epub 2020 Jan 28. PMID: 31994339.3199433910.1111/jcmm.14971PMC7077532

[28] Sartorius K, Sartorius B, Winkler C, et al. The biological and diagnostic role of miRNA’s in hepatocellular carcinoma. Front Biosci (Landmark Ed). 2018 Mar 1;23(9):1701–1720.2929345810.2741/4668

[29] Mizuguchi Y, Takizawa T, Yoshida H, et al. Dysregulated miRNA in progression of hepatocellular carcinoma: a systematic review. Hepatol Res. 2016 Mar;46(5):391–406.2649043810.1111/hepr.12606

[30] Wei S, Liu J, Li X, et al. LncRNA MIR17HG inhibits non-small cell lung cancer by upregulating miR-142-3p to downregulate Bach-1. BMC Pulm Med. 2020 Mar 30;20(1):78.3222854610.1186/s12890-020-1112-3PMC7104535

[31] Jin C, Xiao L, Zhou Z, et al. miR-142-3p suppresses the proliferation, migration and invasion through inhibition of NR2F6 in lung adenocarcinoma. Hum Cell. 2019 Oct;32(4):437–446.3116868910.1007/s13577-019-00258-0

[32] Fabian MR, Sonenberg N, Filipowicz W. Regulation of mRNA translation and stability by microRNAs. Annu Rev Biochem. 2010;79(1):351–379.2053388410.1146/annurev-biochem-060308-103103

[33] Dong H, Song J. miR-142-3p reduces the viability of human cervical cancer cells by negatively regulating the cytoplasmic localization of HMGB1. Exp Ther Med. 2021 Mar;21(3):212.3350070210.3892/etm.2021.9644PMC7818541

The article "Repressing phosphatidylinositol-4,5-bisphosphate 3-kinase catalytic subunit gamma by microRNA-142-3p restrains the progression of hepatocellular carcinoma" was retracted in 2024. Reasons: original data or images not available; unreliable results or conclusions; concerns about the data; concerns about the results or conclusions.

[34] Liu P, Cao F, Sui J, et al. MicroRNA-142-3p inhibits tumorigenesis of colorectal cancer via suppressing the activation of wnt signaling by directly targeting to β-Catenin. Front Oncol. 2021;10:552944.3364389410.3389/fonc.2020.552944PMC7905391

[35] Li Z, Li N, Sun X, et al. FAM98A promotes cancer progression in endometrial carcinoma. Mol Cell Biochem. 2019 Sep;459(1–2):131–139.3111493410.1007/s11010-019-03556-1

[36] Chen J, Bai M, Ning C, et al. Gankyrin facilitates follicle-stimulating hormone-driven ovarian cancer cell proliferation through the PI3K/AKT/HIF-1α/cyclin D1 pathway. Oncogene. 2016 May 12;35(19):2506–2517.2636461610.1038/onc.2015.316

[37] Gao L, Li J, He J, et al. CD90 affects the biological behavior and energy metabolism level of gastric cancer cells by targeting the PI3K/AKT/HIF-1α signaling pathway. Oncol Lett. 2021 Mar;21(3):191.3357493010.3892/ol.2021.12451PMC7816286

[38] Zhang J, Guo H, Zhu JS, et al. Inhibition of phosphoinositide 3-kinase/Akt pathway decreases hypoxia inducible factor-1α expression and increases therapeutic efficacy of paclitaxel in human hypoxic gastric cancer cells. Oncol Lett. 2014 May;7(5):1401–1408.2476514510.3892/ol.2014.1963PMC3997665

[39] Jiao M, Nan KJ. Activation of PI3 kinase/Akt/HIF-1α pathway contributes to hypoxia-induced epithelial-mesenchymal transition and chemoresistance in hepatocellular carcinoma. Int J Oncol. 2012 Feb;40(2):461–468.2192213110.3892/ijo.2011.1197

